# Non-epigenetic function of HDAC8 in regulating breast cancer stem cells by maintaining Notch1 protein stability

**DOI:** 10.18632/oncotarget.6427

**Published:** 2015-11-28

**Authors:** Min-Wu Chao, Po-Chen Chu, Hsiao-Ching Chuang, Fang-Hsiu Shen, Chih-Chien Chou, En-Chi Hsu, Lauren E. Himmel, Han-Li Huang, Huang-Ju Tu, Samuel K. Kulp, Che-Ming Teng, Ching-Shih Chen

**Affiliations:** ^1^ Division of Medicinal Chemistry, College of Pharmacy and Comprehensive Cancer Center, Columbus, Ohio, USA; ^2^ Institute of Pharmacology, College of Medicine, National Taiwan University, Taipei, Taiwan; ^3^ Institute of Biological Chemistry, Academia Sinica, Taipei, Taiwan; ^4^ Department of Veterinary Biosciences, College of Veterinary Medicine, The Ohio State University, Columbus, Ohio, USA

**Keywords:** cancer stem cells, breast cancer, histone deacetylase 8, histone deacetylase inhibitors, Notch1

## Abstract

Here, we report a novel non-epigenetic function of histone deacetylase (HDAC) 8 in activating cancer stem cell (CSC)-like properties in breast cancer cells by enhancing the stability of Notch1 protein. The pan-HDAC inhibitors AR-42 and SAHA, and the class I HDAC inhibitor depsipeptide, suppressed mammosphere formation and other CSC markers by reducing Notch1 expression in MDA-MB-231 and SUM-159 cells. Interrogation of individual class I isoforms (HDAC1–3 and 8) using si/shRNA-mediated knockdown, ectopic expression and/or pharmacological inhibition revealed HDAC8 to be the primary mediator of this drug effect. This suppression of Notch1 in response to HDAC8 inhibition was abrogated by the proteasome inhibitor MG132 and siRNA-induced silencing of Fbwx7, indicating Notch1 suppression occurred through proteasomal degradation. However, co-immunoprecipitation analysis indicated that HDAC8 did not form complexes with Notch1 and HDAC inhibition had no effect on Notch1 acetylation. In a xenograft tumor model, the tumorigenicity of breast cancer cells was decreased by HDAC8 knockdown. These findings suggest the therapeutic potential of HDAC8 inhibition to suppress Notch1 signaling in breast cancer.

## INTRODUCTION

In many types of cancer, a subset of the tumor cell population, called cancer stem cells (CSCs) or tumor-initiating cells, has been linked to tumor initiation, recurrence, chemoresistance, and metastasis [1]. CSCs are characterized by tumorigenic properties and the capacity for self-renewal and differentiation which involve a number of key signaling pathways, including those mediated by Notch [2]. These pathways offer therapeutic opportunities to target CSCs which represent a clinical challenge that must be addressed to achieve optimal patient response [3].

Recent evidence has implicated dysregulated Notch signaling in the maintenance of breast CSCs [4, 5], which may underlie the reported correlation between overexpression of Notch1 or the Notch ligand Jagged-1 and poor prognosis in breast cancer patients [6]. Activation of Notch signaling upregulates a series of target genes, which serve to block cellular differentiation while promoting cell survival and proliferation; thereby promoting a stem-like phenotype in these cells [7]. In addition, dysregulated Notch activity has been reported to lead to a glycolytic switch through activation of the Akt pathway [8] and upregulation of IL-6 expression [9] in breast tumor cells. This mechanistic link between Notch signaling and tumorigenesis was corroborated in mouse models in which the mammary gland-specific activation of Notch caused the formation of papillary tumors [10], and Notch1 inhibition resulted in mammary tumor regression and reduced disease recurrence [11]. Furthermore, in ER + and Her2/neu + breast cancers, drug-resistant phenotypes that emerge following receptor-targeted therapies are believed to be dependent on Notch signaling for continued survival and proliferation [12, 13]. Due to its critical role in cancer stem cell renewal, Notch inhibition has emerged as a viable strategy for cancer stem cell elimination, and several drugs inhibiting various elements of this pathway are in development [14].

Substantial evidence has demonstrated the clinical benefits of HDAC inhibitors as cancer therapeutic agents in both solid tumors and hematological malignancies as a result of their ability to promote differentiation, cell cycle arrest, and apoptosis in cancer cells [15]. The epigenetic effects of HDAC inhibitors can be achieved through multiple mechanisms, including bulk acetylation of lysine residues on the tails of histone proteins, or by blocking the activity of HDACs which act in concert with transcriptional corepressor complexes [16]. Alternatively, HDAC inhibitors might also deacetylate non-histone proteins, such as Hsp90 and p53 [15], which can significantly impact the cellular acetylome by altering protein stability, localization, and/or binding affinity [17]. Recently, it was reported that the pan-HDAC inhibitor abexinostat induced the differentiation of CSCs in breast cancer cell lines exhibiting low expression levels of the long noncoding RNA Xist [18]. Here, we show evidence that, not only pan-HDAC inhibitors, but also a class I HDAC inhibitor, were equally effective in suppressing the CSC population in two triple-negative cancer cell lines, MDA-MB-231 and SUM-159. In the course of our interrogation of the mechanism by which HDAC inhibitors suppress CSC-like properties in breast cancer cells, we obtained evidence that HDAC8, a class I HDAC, plays a pivotal role in maintaining Notch1 protein stability by protecting against Fbw7-mediated proteasomal degradation, independently of its deacetylation activity. The *in vivo* effects of HDAC8 inhibition were demonstrated in a xenograft tumor model in which the incidence of tumor formation from HDAC8-knockdown MDA-MB-231 cells was markedly decreased compared to the parental cell line. These findings may foster new therapeutic strategies for eliminating breast CSCs by inhibiting HDAC8.

## RESULTS

### Suppressive effect of HDAC inhibitors on breast CSCs (BCSCs) is associated with Notch1 downregulation

To shed light onto the mechanistic link between HDAC and BCSCs, we assessed the effects of the pan-HDAC inhibitors AR-42 and SAHA (vorinostat) versus those of the class I HDAC inhibitor depsipeptide (romidepsin) on mammosphere formation, a surrogate measure of CSC expansion [19, 20], in two breast cancer cell lines, MDA-MB-231 and SUM-159. As shown in Figure 1A, these HDAC inhibitors exhibited differential, dose-dependent suppressive effects on mammosphere formation in both cell lines. The effects of HDAC inhibition on BCSCs were also verified by reductions in the CD44^+^/CD24^low^ subpopulation of MDA-MB-231 cells in response to AR-42 and SAHA (Figure 1B). Moreover, Western blot analysis indicated that the HDAC inhibitor-induced suppression of CSC-like properties in MDA-MB-231 cells was associated with the inhibition of Notch1 signaling, as manifested by parallel decreases in the expression levels of Notch1, Notch intracellular domain (NICD), and multiple downstream putative CSC markers, including Nestin, Zeb-1, and BMI-1 (Figure 1C). This HDAC inhibitor-induced downregulation of Notch1 expression was also noted in SUM-159 cells (Figure 1D), indicating that this effect was not a cell line-specific phenomenon.

**Figure 1:** HDAC inhibitors suppress BCSCs, in part, by downregulating Notch1 expression Concentration-dependent effects of AR-42, SAHA, and/or depsipeptide (Depsi) on (**A**) mammosphere formation in MDA-MB-231 and SUM-159 cells, (**B**) the CD44^+^/CD24^low^ subpopulation in MDA-MB-231 cells, and (**C** and **D**) the expression levels of acetyl-histone H3 (Ac-H3), Notch1, NICD, and/or the downstream stemness markers nestin, Zeb-1, and BMI-1 in (C) MDA-MB-231 and (D) SUM-159 cells after 72 h of treatment. Data are expressed as mean ± S.D. (*n* = 6).

### Evidence that HDAC8 is responsible for HDAC inhibitor-induced Notch1 downregulation

The ability of depsipeptide to suppress Notch1 expression suggested that this effect might be mediated through the inhibition of class I HDAC isoforms (HDAC1, 2, 3, and 8). Consequently, we assessed the effect of siRNA-mediated knockdown of individual HDAC isoforms on Notch1 expression in MDA-MB-231 and SUM-159 cells. Knockdown of HDAC 1, 2, 3, and 6, using three different siRNAs for each isoform, individually and in combination, did not appreciably decrease Notch1 expression in either MDA-MB-231 or SUM-159 cells (Figure 2A), which refuted the involvement of any of these isoforms in HDAC inhibitor-mediated Notch1 downregulation.

**Figure 2:** Evidence that HDAC8 is the important isoform for HDAC inhibitor-induced Notch1 downregulation (**A**) Effects of siRNA-mediated knockdown of HDAC1, 2, 3, and 6 on Notch1 expression in MDA-MB-231 and SUM-159 cells. For each HDAC isoform, three different siRNAs, each alone and in combination (Mix), were used. (**B**) Effect of knockdown of HDAC8 by two different shRNAs on the expression of Notch1, HDAC1–3, and the putative CSC markers CD133, CD44, and KLF4 in MDA-MB-231 cells.

In contrast, knockdown of HDAC8 in MDA-MB-231 cells, using two different shRNAs (#71 and #74) that displayed no cross-inhibition of the other three class I HDAC isoforms, led to concomitant decreases in the expression of Notch1 and the CSC markers CD133, CD44 and Kruppel-like factor 4 (KLF4) (Figure 2B). Moreover, this HDAC8 knockdown-mediated inhibition of Notch1 signaling, as shown by reduced expression of Notch 1 and its downstream targets NICD, Nestin, and BMI-1, decreased the abilities of MDA-MB-231 and SUM159 cells to form mammospheres as compared to control cells (Figure 3A). In addition, PCI-34051, a HDAC8-specific inhibitor [21], confirmed that HDAC8-targeted inhibition was sufficient to suppress Notch1 expression and CSC phenotype (Figure 3B). Specifically, exposure of MDA-MB-231 cells to PCI-34051 led to concentration-dependent reductions in Notch 1, Nestin, and BMI-1 expression, and mammosphere formation (Figure 3B), reminiscent of the effects observed with HDAC8 knockdown. In line with the previous report that PCI-34051 did not cause histone acetylation in leukemia cells [21], this drug treatment did not cause an increase, but rather a gradual decrease, in acetyl-histone H3 levels.

**Figure 3:** Knockdown of HDAC8 suppresses CSC phenotype (**A**) Suppressive effect of shRNA-mediated HDAC8 knockdown on the expression levels of Notch1 and its downstream markers NICD, nestin, and BMI-1 (left), and mammosphere formation (right) in MDA-MB-231 and SUM-159 cells. Data are expressed as mean ± S.D. (*n* = 6). (**B**) Concentration-dependent effect of the HDAC8 inhibitor PCI-34051 on the expression levels of Notch1, its downstream markers nestin, and BMI-1, and Ac-H3 (left), and mammosphere formation (right) in MDA-MB-231 cells. Data are expressed as mean ± S.D. (*n* = 6). (**C**) Left, expression profile of Notch1 versus that of HDAC8 in nine different breast cancer cell lines. Right, suppressive effect of HDAC8 knockdown by two different shRNAs on Notch1 expression in T47D cells. 231, MDA-MB-231; 468, MDA-MB-468.

To interrogate the functional relationship between HDAC8 and Notch1, we assessed the protein expression profiles of Notch1 versus HDAC8 in a panel of breast cancer cell lines, including MDA-MB-231, SUM-159, T47D, BT474, HCC1937, MCF-7, SKBR3, MDA-MB-468, and ZR7530 (Figure 3C, left). With the exception of BT474 and MDA-MB-468 cells, HDAC8 expression was positively correlated with that of Notch1, with SUM-159 cells exhibiting the highest abundance of both HDAC8 and Notch1, followed by T47D and MDA-MB-231 cells. In line with the data from MDA-MB-231 and SUM-159 cells, HDAC8 knockdown in T47D cells suppressed Notch1 expression (Figure 3C, right).

The role of HDAC8 in regulating Notch1 expression was further corroborated by the ability of enforced expression of HDAC8 to increase Notch1 levels in MDA-MB-231 and SUM-159 cells. This effect, however, was not shared by the overexpression of HDAC1 or 3 (Figure 4A). Moreover, this effect of HDAC8 on Notch 1 expression was also noted in MDA-MB-468 cells, but was lacking in MCF-7 cells (Figure 4B). These findings reveal apparent cell context-related differences in the regulation of Notch1 expression between MDA-MB-468 and MCF-7 cells, which differ in the functional status of estrogen receptor-α and p53. Importantly, this HDAC8-induced upregulation of Notch1 expression promoted CSC-like phenotype in MDA-MB-231 and SUM-159 cells, as indicated by increased abundance of NICD, the Notch ligand Jagged-1, and the stemness markers Nestin and BMI-1, and mammosphere formation (Figure 4C).

**Figure 4:** Overexpression of HDAC8, but not HDAC1 or 3, increases Notch1 signaling (**A**) Comparison of the effects of the ectopic expression of HDAC1 and 3 versus that of HDAC8 on Notch 1 expression in MDA-MB-231 (upper) and SUM-159 cells. (**B**) Ectopic expression of HDAC8 also increases Notch1 expression in MDA-MB-468 (left), but not in MCF-7 (right) cells. (**C**) Overexpression of HDAC8 activates Notch1 signaling, as manifested by increased expression of Notch, NICD, Jagged 1, nestin, and BMI-1 (left), and increases mammosphere formation (right) in MDA-MB-231 and SUM-159 cells. Data are expressed as mean ± S.D. (*n* = 6).

### HDAC8 inhibition downregulates Notch1 through Fbwx7-dependent protein degradation

Western blot and RT-PCR analyses indicate that the decrease in Notch1 expression after HDAC8 knockdown was mediated at the posttranscriptional level as the abundance of Notch1 mRNA remained unchanged in HDAC8-silenced MDA-MB-231 cells (Figure 5A). This finding refutes a role for the epigenetic repression of *Notch1* gene expression that was reported in valproic acid-treated osteosarcoma cells [22], and is consistent with the cytoplasmic localization of HDAC8 in MDA-MB-231 cells, irrespective of treatment with AR-42 (0.5 μM) (Figure 5B). Equally important, the proteasome inhibitor MG132 protected MDA-MB-231 and SUM-159 cells from the HDAC8 knockdown-induced suppression of Notch1 expression, indicating the involvement of proteasomal degradation in this loss of Notch1 protein (Figure 5C). This premise was corroborated by the ability of HDAC8 shRNA, relative to control, to increase the extent of ubiquitination on Notch1, which was further augmented by MG132 (Figure 5D). As Fbwx7 (aka, Fbw7) is the E3 ligase that plays a central role in the degradation of Notch protein [23], we examined its involvement in HDAC8 knockdown-mediated Notch1 downregulation. The siRNA-mediated silencing of Fbwx7 increased Notch1 expression in MDA-MB-231 cells (Figure 5E, left) and, more importantly, protected cells from the suppressive effect of HDAC8 knockdown on Notch1 expression (right). It is interesting to note that HDAC8 knockdown led to reduced expression levels of Fbwx7, of which the underlying mechanism warrants investigation.

**Figure 5:** HDAC8 inhibition facilitates Fbwx7-dependent degradation of Notch1 (**A**) Western blot (upper) and RT-PCR (lower) analyses of the effect of HDAC8 knockdown on the protein and mRNA expression, respectively, of Notch1 in MDA-MB-231 cells. (**B**) Left, Western blot analysis of the cellular distribution of HDAC8 in MDA-MB-231 cells after 72 h treatment with DMSO control (−) or 0.5 μM AR-42 (+). Right, immunocytochemical analyses of the cellular distribution of HDAC8 in untreated MDA-MB-231 cells. Scale bar, 20 μm. (**C**) The proteasome inhibitor MG-132 (2.5 μM, 24 h) protected against HDAC8 knockdown-facilitated suppression of Notch1 expression in MDA-MB-231 and SUM-159 cells. (**D**) Co-immunoprecipitation analysis of the effect of MG-132 on Notch1 ubiquitination in MDA-MB-231 cells in the presence or absence of shRNA-mediated HDAC8 knockdown. (**E**) The silencing of Fbwx7 increased Notch1 expression (left) and protected against HDAC8 knockdown-induced downregulation of Notch1 (right) in MDA-MB-231 cells. (**F**) The GSK3β inhibitor SB216763 (left) and the CK2 inhibitor DMAT (right) did not protect against AR-42-facilitated suppression of Notch1 expression in MDA-MB-231.

Moreover, it is well documented that E3 ligase-mediated ubiquitination is preceded by substrate phosphorylation [24]. As glycogen synthase kinase (GSK) 3β [25, 26] and casein kinase (CK) 2 [27] have been reported to inhibit Notch1 stability and/or transcriptional activity, we examined their roles in mediating AR-42-facilitated Notch1 degradation by co-treating MDA-MB-231 cells with AR-42 and the respective kinase inhibitors SB216763 or 2-dimethylamino-4, 5, 6, 7-tetrabromo-1H-benzimidazole (DMAT). Neither compound reversed the suppressive effect of AR-42 on Notch1 expression (Figure 5F), suggesting the involvement of another kinase in AR-42-induced downregulation of Notch1 expression.

### Evidence that HDAC8 does not bind Notch1

In addition to catalyzing the deacetylation of histone and nonhistone substrates [28], HDAC8 has also been reported to bind and protect human ever-shorter telomerases 1B (hEST1B) protein from ubiquitin-facilitated degradation independently of its deacetylase activity [29]. Based on this finding, we rationalized that HDAC8 might increase Notch1 protein stability in a similar fashion through complex formation. Accordingly, we examined the physical interaction of endogenous HDAC8 with Notch1 in MDA-MB-231 cells via co-immunoprecipitation. No appreciable HDAC8 was detected in association with immunoprecipiated Notch1, indicating that HDAC8 did not form complexes with Notch1 (Figure 6A). Furthermore, we determined that the ability of HDAC8 to stabilize Notch1 may be independent of its effect on protein acetylation. Notch1 (molecular mass, 130 kD) immunoprecipitated from the lysates of AR-42-treated MDA-MB-231 cells exhibited no appreciable level of acetylation relative to that of control (Figure 6B).

**Figure 6:** Evidence that HDAC8 does not bind Notch1 (**A**) Co-immunoprecipitation analysis of the presence of endogenous Notch1-HDAC8 complexes in MDA-MB-231 cells. (**B**) Co-immunoprecipitation analysis of the effect of AR-42 (0.25 μM, 48 h) versus DMSO control on the acetylation level of Notch1 in MDA-MB-231 cells. *molecular weight of Notch1.

### HDAC8 contributes to breast tumorigenicity *in vivo*

As CSCs are characterized by their capacity to form tumors from low cell numbers, we assessed the effect of HDAC8 knockdown on tumor-initiation by MDA-MB-231 cells. Female NOD/SCID mice were injected bilaterally into mammary fat pads with 50, 000 MDA-MB-231 cells stably expressing HDAC8 shRNA (HDAC8^KD^; Figure 7A, left) on one side and an equal number of control (Void) MDA-MB-231 cells on the opposite side. At one week post-injection, 100% of mice had tumors generated from the control Void cells, while only 50% of mice had HDAC^KD^ tumors. From 2–4 weeks post-injection, the difference in tumor-free incidence between HDAC8^KD^ and control MDA-MB-231 tumors remained at 30% for the rest of the study (*P* = 0.0118; log-rank test) (right). Moreover, the HDAC8^KD^ tumors grew at a slower rate than the control tumors, but this difference was not statistically significant (Figure 7B).

**Figure 7:** HDAC8 knockdown suppresses tumor-initiating ability of BCSCs *in vivo* (**A**) Left, Western blot analysis of HDAC8 and Notch1 expression in the stable clone of HDAC8 knockdown (HDAC8^KD^) MDA-MB-231 cells. Right, effect of HDAC8 knockdown on tumor-initiating ability of MDA-MB-231 cells. The stable HDAC8^KD^ MDA-MB-231 clone (#74) and control MDA-MB-231 cells (Void) were injected (50,000 cells/injection) into contralateral inguinal mammary fat pads of NOD/SCID mice (*n* = 10), and tumor incidence was monitored over 28 days. (**B**) Effect of HDAC8 knockdown on MDA-MB-231 xenograft tumor growth in the same experiment. Data are expressed as means ± S.D.

## DISCUSSION

In this study, we report a novel non-epigenetic function of HDAC8 in regulating CSC-like properties in breast cancer cells by maintaining the stability of Notch1 protein, which might underlie the reported ability of HDAC inhibitors to activate Notch1 signaling in cancer cells. Although HDAC8 is the best mechanistically and structurally characterized HDAC isoform, its biological role remains elusive, because its reported functions vary with its intracellular location in a cell type- and context-specific manner [review: [28]]. In contrast to other class I HDACs, HDAC8 does not require additional protein cofactors to catalyze deacetylation [28], and has few identified non-histone substrates, which include heat shock protein (Hsp) 20 [30], estrogen-related receptor (ERR)α [31], and the core cohesin component SMC3 [32].

A tumorigenic role for HDAC8 has been suggested by its high expression levels in childhood neuroblastoma [33] and hepatocellular carcinoma [34], which warrants attention. Mechanistically, HDAC8 might facilitate tumorigenesis through distinct mechanisms at the epigenetic and/or cellular level in a cell type-specific manner. For example, HDAC8 has been reported to form corepressor complexes with Stat3 to repress the proapoptotic target gene *BMF* in colon cancer cells [35], and to activate Jak2/Stat signaling through epigenetic repression of *SOCS1* and *SOCS3* genes in K562 and HEL erythroleukemia cells [36]. Data from the present and other studies have demonstrated a niche role of cytoplasmic HDAC8 in determining the fate of non-histone substrates. We present evidence that HDAC8 protects Notch1 from Fbwx7-facilitated protein degradation in breast cancer cells, which is reminiscent of the protective effect of HDAC8 on hEST1B protein stability in HeLa cells [29]. As HDAC8 did not bind to or cause acetylation of Notch1, it is plausible that this protective effect might be associated with the ability of HDAC8 to inhibit Fbwx7 activity, which is currently under investigation.

In addition to HDAC8, HDAC3 has also been reported to participate in the self-renewal of liver CSCs through histone modifications [37]. Besides deacetylase activity on core histones, HDAC3 also shows biological functions beyond transcriptional repression [38]. The putative role of HDAC3 in regulating CSCs is supported by our finding that the class I HDAC inhibitor MS-275, which is deficient in HDAC8 inhibitory activity, suppressed mammosphere formation in breast cancer cell lines (data not shown). From a mechanistic perspective, the potential interplay between HDAC8 and HDAC3 in mediating the non-epigenetic versus epigenetic effects of HDAC inhibitors on CSCs warrants attention.

In this study, we provide evidence of a novel role for HDAC8 in maintaining Notch1 protein stability in breast cancer cells by limiting Fbwx7-facilitated proteasomal degradation, leading to the promotion of CSC phenotype. These findings suggest that the inhibition of HDAC8 may represent a therapeutic approach for suppressing the breast CSC subpopulation.

## MATERIALS AND METHODS

### Cell lines and biochemical agents

MDA-MB-231, MCF-7, MDA-MB-468, BT474, T47D, HCC1937, SKBR3 and ZR7530 breast cancer cell lines were purchased from American Type Culture Collection (Manassas, VA) and cultured in DMEM, F12/MEM or RPMI 1640 medium (Life Technologies; Grand Island, NY) supplemented with 10% fetal bovine serum (Life Technologies), 100 U/ml penicillin, 100 μg/ml streptomycin and 50 μg/ml gentamycin B (Life Technologies). SUM159 cells were purchased from Asterand Biosciences (Detroit, MI) and cultured in Ham's F-12 (Life Technologies) supplemented with 5% fetal bovine serum, 5 μg/ml insulin, 1 μg/ml hydrocortisone, 100 U/ml penicillin, 100 μg/ml streptomycin and 50 μg/ml gentamycin B. All cells were cultured at 37°C in a humidified incubator containing 5% CO_2_, and were used in fewer than 6 months of continuous passage. AR-42 was obtained from Arno Therapeutics (Flemington, NJ). Vorinostat and romidepsin (referred to as SAHA and depsipeptide, respectively) were purchased from ChemieTek (Indianapolis, IN). PCI-34051 was purchased from Cayman Chemical (Ann Arbor, MI) and MG132 was obtained from Sigma-Aldrich (St. Louis, MO). Antibodies against various proteins were from the following sources: CD44, KLF4, Notch1, NICD, BMI-1, Zeb-1, Jagged 1, HDAC3, and acetyl-lysine, Cell Signaling Technology (Beverly, MA); HDAC1, 2, and 8 and GAPDH, Santa Cruz Biotechnology (Santa Cruz, CA); Nestin, BD Biosciences (San Jose, CA); conjugated CD44 and CD24, BD (Franklin Lakes, NJ); CD133, Proteintech Group (Chicago, IL); Fbw7, Abcam (Cambridge, MA); acetyl-histone H3, Millipore (Billerica, MA); horse radish peroxidase-conjugated anti-mouse IgG and anti-rabbit IgG, Jackson ImmunoResearch Laboratories (West Grove, PA).

### Mammosphere formation assay

Five hundred SUM159 cells/well and 1, 000 MDA-MB-231 cells/well were seeded onto ultra-low attachment 24-well flat bottom plates in serum-free culture medium (MammoCult^™^, STEMCELL Technologies; Vancouver, BC, Canada). Cells were then treated with the indicated compounds for 7 days, after which the numbers of mammospheres were counted at 100X magnification.

### Flow cytometry

The CD44^+^/CD24^low^ subpopulations of breast cancer cells were analyzed by flow cytometry. Treated cells were harvested and then incubated with specific FITC- or phycoerythrin-conjugated monoclonal antibodies against CD44 and CD24 on ice in the dark for 30 min. Cells were washed with BSA-PBS and the pellets were collected and suspended in PBS. Cells were sorted and analyzed using a FACSCalibur (BD Biosciences) flow cytometer.

### Western blotting

Cell pellets were lysed in RIPA lysis buffer and sonicated. The protein concentration in each sample was determined using the BCA Protein Assay kit (Thermo Fisher Scientific, Waltham, MA). An equal amount of protein from each sample was loaded per lane, separated by SDS-PAGE, and then transferred onto nitrocellulose membranes. Transferred membranes were blocked with 5% non-fat milk for 1 h and then incubated with primary antibodies overnight at 4°C. On the next day, membranes were washed with TBST and incubated with the corresponding secondary antibodies for 1 h at room temperature. Chemiluminescence Reagent Plus (Perkin-Elmer; Waltham, MA) was used to detect signals.

### General and lentivirus transfection

Cells were transfected with plasmids and siRNAs using Lipofectamine 2000 (Life Technologies) according to the manufacturers’ instructions. The plasmids and siRNA used in this study and their sources were as follows: pCDNA3.1, Flag-HDAC1, 3 and 8 (Addgene, Cambridge, MA); HDAC1, and 8 siRNA (Life Technologies); HDAC2, 3, and 6 siRNA (OriGene, Rockville, MD). Lentivirial plasmids were cotransfected with Addgene 3rd Generation Packaging Systems (pMDLg/pRRE [#12251], pRSV-Rev [#12253] and pMD2.G [#12259]) in 293T cells following a standard calcium phosphate transfection procedure. Viral particles were used for infection of target cells and stable cells were selected by exposure to puromycin for one week. pLAS.Void (negative control) and HDAC8 shRNA were obtained from Academia Sinica (Taipei, Taiwan). The HDAC8 expression plasmid was constructed in pLenti CMVTRE3G Puro DEST (w811–1) vector (Addgene) by LR reaction after cloning HDAC8 cDNA into the pENTR noccDB (w48–1) entry vector (Addgene).

### RT-PCR analysis

Total RNA was isolated from cells with TRIzol (Thermo Fisher Scientific) according to the manufacturer's protocol. One μg RNA from each sample was reverse-transcribed into cDNA using the iScript^™^ cDNA Synthesis Kit (Bio-Rad; Hercules, CA), which was then mixed with buffer, dNTP, polymerase (Bio-Rad; Hercules, CA), ddH_2_0 and primers. The resulting PCR products were separated by electrophoresis in a 1% agarose gel. The following primers were used: HDAC8, forward: 5′-GATCAGAGGAGCAGGAACTG-3′, reverse: 5′-CTGCTTATGCAGTGCATATGC-3′; Notch1, forward: 5′-ATCGGGCACCTGAACGTGGCG-3′, reverse: 5′-CACGTCTGCCTGGCTCGGCTC-3′; GAPDH, forward: 5′-CGACCACTTTGCAAGCTCA-3′, reverse: 5′-AGGGGTCTACATGGCAACTG-3′.

### Immunoprecipitation

Cells were harvested, incubated in IP lysis buffer (20 mM Tris-HCl pH 7.5, 150 mM NaCl, 1% Triton X-100) for 30 min on ice, and then sonicated (3 times for 10 sec each). After centrifugation, the supernatants were collected from each sample and then pre-cleared by incubation with 10 μl protein A/G agarose beads at 4°C for 1 h with rocking. After removal of the protein A/G beads by centrifugation, protein content in each sample was measured and aliquots containing 1500 μg of protein were incubated with primary antibodies overnight at 4°C with rocking, followed by 20 μl protein A/G agarose beads for 2 h at 4°C. The immunoprecipitates were washed with IP lysis buffer, collected by centrifugation, and resuspended in 2X sample buffer for analysis by immunoblotting.

### Immunofluorescence

Cells were seeded onto round cover glasses in 6-well culture plates. After treatments, the cells were fixed with 4% paraformaldehyde (in PBS) for 20 min, and then permeabilized with 0.2% Triton X-100 (in PBS) for 10 min. The cells were blocked with 1% BSA in PBS for 1 h, and then incubated with primary antibody overnight at 4°C. After washing with PBS, cells were incubated with secondary antibody for 2 h at room temperature. The cover glasses were mounted with Vectashield mounting medium (Vector Laboratories, UK) containing 4′,6-diamidino-2-phenylindole (DAPI) for nuclear staining. Images were obtained with an Olympus FV1000 confocal microscope (Olympus Corp., Japan).

### Animal study

Female NOD/SCID mice (NOD.CB17-*Prkdc^scid^*/NCrHsd; 5–6 weeks of age; Harlan, Indianapolis, IN) were group-housed under constant photoperiod (12 hours light: 12 hours dark) with *ad libitum* access to sterilized food and water. All experimental procedures were done according to protocols approved by The Ohio State University Institutional Animal Care and Use Committee. To assess the role of HDAC8 in tumor initiation *in vivo*, HDAC8^KD^ cells (MDA-MB-231 cells stably expressing HDAC8 shRNA) were injected into the left inguinal mammary fat pads of female NOD/SCID mice (50, 000 cells/0.1 ml, in Matrigel [BD Biosciences]). An equal number of MDA-MB-231 cells expressing the pLAS Void plasmid (Void) were injected into the contralateral mammary gland to serve as negative control. Tumors were measured with calipers and the volumes were calculated using *V =* 1/2 (width^2^ × length).

### Statistical analysis

*In vitro* experiments were performed at least three times and data are presented as means ± SD. Group means were compared using one-way ANOVA followed by Student's *t* tests. For the *in vivo* experiments, differences in tumor incidence and tumor volume were analyzed by log-rank test and Student's *t* test, respectively. Differences were considered significant at *P* < 0.05.
